The article "Perceived family relationships and social participation through sports of urban older adults living alone: An analysis of the mediating effect of self-respect levels" was published in 2023. Journal: Front Public Health.

# Perceived family relationships and social participation through sports of urban older adults living alone: An analysis of the mediating effect of self-respect levels

**DOI:** 10.3389/fpubh.2023.1095302

**Published:** 2023-03-30

**Authors:** Rong Zhou, Jinghang Cui, Xingxing Yin

**Affiliations:** ^1^College of Philosophy, Law and Political Science, Shanghai Normal University, Shanghai, China; ^2^College of Professional Studies, Northeastern University, Boston, MA, United States; ^3^School of Social Development, East China Normal University, Shanghai, China

**Keywords:** family relationships, social participation through sports (SPS), self-respect level, the mediating effect, sports, urban older adults living alone (UOALA)

## Abstract

**Introduction:**

The perception of good family relationship is an important factor to promote social participation through sports of older adults living alone. This study explores the influence of perceived family relationship on sports sociability and its group differences, and then discusses the mediating effect of self-respect.

**Methods:**

Based on the survey data of 2,801 older adults living alone in Chengdu, Shanghai, Guangzhou, Hohhot, and Dalian, the quantitative index of their “activeness in social participation through sports” was constructed. The OLS model, the Ologit model, the instrumental variable method and the mediating effect were used to explore the influence mechanism of perceived family relationships of urban older adults living alone on their sport participation.

**Results:**

The results demonstrate that: (1) Older adults 's activeness in sport participation in China is generally at a low level; (2) perceived family relationships have an impact on activeness in sport participation, i.e. positive family relationships will increase their activeness in sport participation, and there are evident gender differences in this tendency; (3) there are regional differences in the activeness in SPS among the older adults living alone in urban areas, and perceived family relationships in first-tier and second-tier cities have a more significant impact on their activeness in sport participation; (4) the mediating effect analysis shows that perceived family relationships can indirectly promote urban old adults' activeness in sport participation through the reconstruction of their self-respect, and this is more pronounced in women.

**Discussion:**

Therefore, the important role of families cannot be ignored in promoting sport participation of the older adults.

## 1. Introduction

Aging has become an irreversible trend in China's population structure. According to the seventh Chinese census, by the end of 2020, China's population aged 65 and above has reached 191 million, accounting for 13.50% of the total population, approaching the 14% mark which leads to a deep aging society (1). In addition, according to the 1% National Population Sample Survey in 2015, the proportion of single-person households in China was 15.75%, an increase of 4.29% over 2000 (2). With the deepening development of the aging, the social understanding of caring for older adults living alone is no longer based on standardized data research but focused on its social impact.

According to the activity theory, socializing in old age is the key to achieving longevity and mental health, and keep positive interaction with society are more likely to achieve a “successful old age” (3). As early as in the 1990s, Putnam et al. (4) proposed that sports participation is an activity with social attributes as individuals expanded their interpersonal network in the process of building up their strength. Sirven and Debrand (5), Singh and Misra (6) pointed out that the social participation of older adults has significantly contributed to the improvement of their health, and social activities, especially community-based sports, correlate strongly with reducing perceived depression and emotional impairment. Empirical research in China also shows that participation in social activities has a significant impact on the activities of daily living and the risk of death of older adults, and plays an important role in alleviating the degradation of physical and psychological functions and maintaining physical and mental health (7). However, Warner et al. (8) suggested that loneliness peaks in old age, largely due to the empty nest syndrome, a phenomenon in which parents experience negative feelings when children leave home. New dependence and support relationships are constantly reconstructed in daily social inter-action through physical exercise (9). In addition to elaborating from the perspectives of role involvement, social interaction, and functioning (10, 11), affected by the special cultural background and historical national conditions, East Asia is more accustomed to the family to explain various social problems in old age. Family relationship is the core of East Asian cultural tradition, so it is more important to analyze the social behavior of the older adults in sports from the family.

The research significance of this paper is as follows: First, with the change of Chinese family population structure, the scale of older adults living alone continues to rise. Compared with the previous studies which took ordinary older adults as the object, this study focuses on this kind of older adults living alone. Second, rather than using the previous research framework that focuses on the impact of individual differences on sports behavior in old age, this paper attempts to put older adults in the family network based on individual differences to test whether the impact of family relationships on SPS exists (and if it does, how much it is and what are the nature and differences). Third, through what factors do perceived family relationships have an impact on older adults' activeness in SPS? That means an empirical data exploration of the logical relationship between the two. At present, there is no empirical research on this issue, so it cannot fully reflect the effect of perceived family relationship on SPS in the older adults. By introducing the level of self-respect as a mediating variable, this paper makes in-depth discussions on the effect mechanism between the two to find possible solutions to various social problems caused by the increasingly severe aging problem from the traditional family perspective.

So, how to promote SPS of the older adults living alone in cities? Glass et al. pointed out that family relationships have a significant impact on psychological wellbeing at all stages of life (11). Katz (12) further found that a high level of psychological wellbeing is directly related to the overall living conditions of the older group, while family relationships work as a regulator of individual and external risks and can magnify or reduce the impact of external social risks on subjective wellbeing. Silverstein and Bengtson (13) further pointed out that intergenerational solidarity was conducive to physical and mental health and social adaptation in older adults, and can promote their social integration. As the main source of social support for older adults, family relationships may have an important impact on the SPS of older adults living alone. Therefore, this paper puts forward research hypothesis 1:

**H1:** Other things being equal, perceived family relationships have a positive impact on UOALA's SPS.

Without the comparison of gender heterogeneity, it will be difficult to deeply understand the group segmentation of SPS. Due to the combined effects of genes, physiological function and lifestyle, the life expectancy of women is usually higher than that of men (14), and the negative impact of the loss of a spouse makes a woman more dependent on her family (15). Spesivtseva (16) found that family relationships were closely related to self-confidence, and the parent-child relationship was the main factor in female older adults' self-cognition of the social significance and social role, having an important impact on social behavior. Women's physiological gender and social gender are often described as having perceptual and dependent characteristics, so the special obstacles in the way of their sports participation may come from sociocultural and individual aspects (17). When families give emotional support to help them rebuild their sense of identity, their activeness in SPS will be higher. Therefore, this paper puts forward research hypothesis 2:

**H2:** Other things being equal, perceived family relationships have a greater impact on the SPS of female older adults living alone in urban areas.

So, how do family relationships affect UOALA's SPS? Bandura (18) held that self-efficacy was the core factor affecting the direction, intensity and persistence of individual social behavior. SPS is a selective social behavior and its formation is restricted by social construction and individual psychological state. In addition to instrumental support in terms of economy, labor and emotion, intergenerational support will also have an impact on social interaction, values and structural norms (19). Individuals in old age associate secure family attachment more closely with positive self-representation, and high levels of self-respect can help older adults living alone deal with emotions more rationally and engage in social interactions more actively. In other words, if individuals perceive that they are cared for and respected in their family relationships, then this connection can dampen the stress response, reduce stress levels, and improve social participation (20). Therefore, family is an important environmental factor affecting the level of individual self-respect, the relationship between family function and individual self-respect has cross-cultural consistency, harmonious family relations can promote the development of individual self-awareness (21). Li's (22) research also confirmed that children's respect and good care have positive effects on their parents, such as strengthening self-respect and reducing loneliness. Positive family relationships can help individuals rely on the “safe base” provided by their families, thus supporting them in exploring themselves and improving their self-respect (23). As an important indicator of self-conception, self-respect shapes the sense of self-worth, and further affects the social behavior of individuals (24). Stable attachments formed between older adults living alone and other family members provide a “safe base” for individuals to develop themselves, especially their sense of self-respect, thus promoting their sports social initiative. Therefore, this paper puts forward research hypothesis 3:

**H3:** Positive family relationships increase UOALA's activeness in SPS by improving their self-respect.

## 2. Materials and methods

### 2.1. Samples and data sources

The data used in this paper come from the “Research on the Home-Based Care System of Chinese Urban Older Adults in the Next Decade,” a major project of National Social Science Fund funded by the government, which was carried out in Shanghai, Guangzhou, Chengdu, Hohhot and Dalian in 2015–2016.

The choice of survey sites was based on the following considerations: First, economic and geographical factors. The level of social and economic development and the stage of development jointly determine the development level of sports (25). The development of sports in China has distinct regional characteristics. The regional economy plays a great promoting role in the development of mass sports, and there is a huge economic gap between the eastern and western regions. Therefore, the research group chose eastern cities such as Shanghai, Guangzhou and Dalian and western cities such as Hohhot and Chengdu for data collection.

Second, the administrative rank of cities. Sports policies have a direct impact on sports development (26). Affected by the differences in the administrative rank of cities, sports policies are different in terms of levels, objectives, quantity, contents and so on. Therefore, the research group comprehensively chose Shanghai (a municipality directly under the Central Government, provincial level), Guangzhou, Chengdu, Hohhot (prefecture-level and provincial capital cities) and Dalian (prefecture-level and non-provincial capital cities) as the survey sites.

Third, the aging degree of the urban population. The research focuses on UOALA, so the aging degree of the population in their city is the basic information to be considered in the choice of survey sites. In 2015, the five cities belonged to different subtypes of an aging society, so they were selected as the survey sites.

The method of four-stage random sampling was used to select local older adults living alone according to the “administrative district, street, neighborhood and household” they belong to in the five cities. The subjects of this paper are older adults living alone in the survey sites during the survey (by “living alone,” we mean “sleeping alone at night”). The sample data were collected strictly according to the four-stage random sampling method. The first stage: four administrative districts were randomly selected in each city (if the number of administrative districts under the jurisdiction of the surveyed city was equal to or <4, all administrative districts were selected). The second stage: in each selected administrative district, two streets were randomly selected from the streets under its jurisdiction. The third stage: in each selected street, two neighborhoods were randomly selected from all the neighborhoods under its jurisdiction. The fourth stage, 50 older adults living alone were selected according to the house number at a regular interval. If a neighborhood had <50 older adults living alone, the difference would be made up from other neighborhoods on the same street. If the total number of older adults living alone in a selected street was <100, all the eligible subjects in the street would be investigated according to the requirements of cluster sampling.

In order to improve the quality of data collection, we designed a “short questionnaire” and a “long questionnaire” according to the cognitive abilities of the respondents. The “short questionnaire” was numbered the same way as the “long questionnaire,” except that the contents of the former (13 pages) were shorter than that of the latter (24 pages). Thus, the short one was suitable for older adults with low cognitive functions. The scale in the preliminary questionnaire was used to assess cognitive functioning in the subjects (out of 10, with higher scores indicating better cognitive test performance). If the total score reached 6 or above, then the long questionnaire was assigned to the subject; if the total score was at or below 5, the short questionnaire was used. The long questionnaire covered all the questions in the short one. This paper uses the data from the long questionnaire. After data review and supplementary investigation, a total of 2,801 samples were obtained using the long questionnaire, including 429 in Chengdu, 587 in Hohhot, 593 in Dalian, 472 in Guangzhou and 720 in Shanghai. The contents of the survey included their basic information, the situation of their children, occupational income, health, life care, housing, participation in sports and cultural activities, social support and so on. It should be noted that this survey is a cross-sectional survey, not a continuous follow-up, so the age classification in the empirical analysis is a category variable, not a time cohort data.

### 2.2. Model setting and variable measurement

Based on the hypotheses, this study investigated the relationship between UOALA's SPS and their perceived family relationships, and thus the following model:


$$\begin{array}{l} \text{so}{\text{c}}_{\text{i}}=\beta_{\text{0}}+\beta_{\text{1}}\text{fa}{\text{m}}_{\text{i}}+\gamma X_{\text{i}}+\varepsilon \end{array}$$

To examine the mediating effect of self-respect level, the Baron and Kenny method for testing mediation hypotheses was used. (1) As verified above, the control variables have been substituted to run a regression of perceived family relationships to test the effect of perceived family relationships on SPS; (2) Test the effect of perceived family relationships on self-respect levels. If the coefficient of perceived family relationships is significantly positive, it means a positive correlation exists between perceived family relationships and the self-respect level of older adults; (3) Add the mediating variable of self-respect levels to step (1). If the mediating variable has a significant effect while the coefficient of perceived family relationships becomes smaller than in step (1) with a decline in its significance, it means that the level of self-respect of UOALA has a partial or full mediating effect. Based on the above analysis, the test model was set as follows.

Step 1: test whether perceived family relationships affect SPS.

$$\begin{array}{l} \text{so}{\text{c}}_{\text{i}}=\beta_{\text{0}}+\beta_{\text{1}}\text{fa}{\text{m}}_{\text{i}}+\gamma X_{\text{i}}+\varepsilon \end{array}$$

Step 2: test whether perceived family relationships affect self-respect levels.

$$\begin{array}{l} \text{fa}{\text{m}}_{\text{i}}=\beta_{\text{2}}+\beta_{\text{3}}\text{r}esp_{\text{i}}+\gamma X_{\text{i}}+\varepsilon \end{array}$$

Step 3: introduce perceived family relationships and self-respect level variables into the model simultaneously.

$$\begin{array}{l} \text{so}{\text{c}}_{\text{i}}=\beta_{\text{4}}+\beta_{\text{5}}\text{fa}{\text{m}}_{\text{i}}+\beta_{\text{6}}\text{r}esp_{\text{i}}+\gamma X_{\text{i}}+\varepsilon \end{array}$$

where *soc* refers to the frequency of the subjects' SPS, *fam* represents perceived family relationships, *X* represents other control variables, and ε represents a stochastic disturbance term.

The predicted variable is social participation through sports (*soc*). The study of Yang and Wang (27) suggested that unlike the youth's socialization through work, socialization in old age is a mode of behavior that achieves communication and resource sharing at the personal and social levels in daily life, satisfying the needs of all parties while realizing their values, and conceptually, it should include all activities that are beneficial to society and the development of older adults themselves. Group sports activities are the most common form of SPS in the daily life of older adults. Therefore, this paper defines the “SPS in old age” as the communication and interaction of older adults in the process of participating in group sports activities. Various types of senior activity centers at the neighborhood level have assumed the organization of senior sports activities tangibly and become the base station for emotional connections (28). In response to the bottlenecks of empirical research, such as the complex types of sports and social activities in old age, different frequencies, and the difficulty of statistics, and combined with the results of data screening in the database used, this paper constructs the index of “SPS” to comprehensively evaluate the SPS of older adults living alone in urban areas by counting their participation in community or resident activity centers, senior activity rooms or centers, community cultural centers or cultural rooms, various types of senior schools, outdoor or indoor fitness spots. By counting the participation in community or resident activity centers, senior citizen activity rooms or centers, community cultural centers or cultural rooms, various senior citizen schools, and outdoor or indoor fitness spots, we evaluated the degree of their social activity in sports. According to our survey, the mean value of respondents' scores was 0.897, and the frequency of the subjects' SPS was <1, which indicated that the group's activeness in SPS was at a low level.

The core predicted variable is the perceived family relationship (*fam*), which refers to the state of the relationship between family members, indicating the closeness and cohesiveness in a family. In this definition, family harmony is more about the respondents' subjective perceptions. Therefore, the assessment was based on the respondents' answers to the question “How good is the relationship between you and your family,” i.e., “not good or not very good = 1, average = 2, good or very good = 3,” and the higher the score, the better the family relationship.

In addition, according to the previous literature, there is an evident gap between urban and rural areas in older adults' social participation rates. Specifically, the social participation rate of urban older adults is much higher than that of the rural older adults. Although all of the respondents lived in urban areas during the survey, some of them with rural residency might maintain their original lifestyles due to the influence of their habits and mindsets, which had an impact on their activeness in SPS. In addition, studies have shown that educational level and personal comprehensive quality have a positive effect on SPS, because self-confidence makes older adults more willing to engage in social activities (29). Unstable marital life can keep older adults away from social participation, and thus married older adults are more active in social participation than unmarried, divorced, or widowed ones. Therefore, the control variables in this study encompassed demographic factors that might have an impact, such as age (*age*), residency (*res*), education levels (*edu*), and marital status (*mar*).

Economic conditions were measured by average monthly income (inc), and previous studies have shown that the use of personal income by older adults implies good economic conditions (30). A solid financial foundation is a prerequisite element for older adults to engage in sporting activities, and thus the income level directly affects the activity engagement of older adults. Low-income older adults usually belong to a low-activity group, while high-income older adults are more likely to be high-activity individuals. Similarly, health status is an important indicator of older adults' SPS, as good health is essential for them to engage in various activities and social life. Although self-reported health is a subjective evaluation, it has high reliability (31). Therefore, this paper examines the degree of health mainly in terms of both subjective and objective aspects, i.e., self-reported health (heal) and the number of confirmed illnesses (ill, the total of the types of illnesses described by older adults). Moreover, the number of children is another relevant factor. In the process of modernization, family security is internal and fundamental. The resilience, flexibility, solidarity and tension of traditional family intergenerational relationships are closely related to the number of children. Therefore, the number of children needs to be controlled. See Table 1 for specific assignments.

**Table 1:** Descriptive statistics.

**Variables**	**Options**	**Sample size**	**Average value**	**Standard deviation**
*soc*	The total frequency of respondents' SPS	2,739	0.897	1.270
*fam*	Not good or not very good = 1, average = 2, good or very good = 3	2,675	4.321	0.799
*age*	Filled in by respondents	2,801	78.470	5.358
*resi*	Non-rural residency = 1, rural residency = 0	2,779	0.951	0.215
*edu*	Illiteracy or no schooling = 1, primary education = 2, primary education = 3, upper secondary education = 4, post-secondary non-tertiary education = 5, tertiary education = 6	2,776	2.634	1.319
*mar*	Never married = 1, married = 2, divorced = 3, widowed = 4	2,763	3.539	0.875
*inc*	500 yuan or less = 1; 500–999 yuan = 2; 1,000–1,499 yuan = 3; 1,500–1,999 yuan = 4; 2,000–2,499 yuan = 5; 2,500–2,999 yuan = 6; 3,000–3,999 yuan = 7; 4,000–4,999 yuan = 8; 5,000 yuan and above = 9	2,789	5.027	1.858
*heal*	Very good = 1; good = 2; average = 3; not good = 4; bad = 5	2,706	2.967	1.060
*ill*	Total types of illnesses described	2,779	1.692	1.214
*resp*	With great difficulty = 1; with some difficulty = 2; with no difficulty = 3	2,106	2.461	0.678
*child*	Number of children (living children, including children recognized by law such as adopted ones)	2,715	2.70	1.28
*prox*	The same neighborhood = 1, the same street or town, but different neighborhoods = 2, the same city (district or county), but different streets or towns = 3, the same province (autonomous region, municipality directly under the Central Government), but different cities (districts, counties) = 5, different provinces (autonomous regions, municipalities directly under the Central Government) in the Chinese mainland = 6, outside the Chinese mainland = 7	2,600	2.74	0.78

## 3. Results

### 3.1. Benchmarking regression

According to the research hypotheses, the effects of perceived family relationships on the SPS of UOALA are shown in Table 2. The first three models were the estimates calculated by OLS models, and the robustness of the last three models was tested by Ologit regression models. The results show that the coefficient of perceived family relationships (0.170) is evidently positive at the 0.01 level, with factors such as demographic characteristics and the number of children being controlled. This indicates that a significant positive correlation exists between perceived family relationships and the SPS of UOALA.

**Table 2:** Effects of perceived family relationships on SPS of older adults living alone.

	**Benchmarking regression**						**Robustness test**	
	**OLS**			**Ologit**			**OLS**	**Ologit**
	**(1)**	**(2)**	**(3)**	**(4)**	**(5)**	**(6)**	**(7)**	**(8)**
	**Full sample**	**Male**	**Female**	**Full sample**	**Male**	**Female**	**Full sample**	**Full sample**
*fam*	0.170^***^ (−0.058)	0.202^**^ (−0.102)	0.156^**^ (−0.07)	0.117^**^ (−0.056)	0.094 (−0.099)	0.123^*^ (−0.069)	0.149^***^ (−0.044)	0.234^***^ (−0.079)
*age*	−0.043^***^ (−0.005)	−0.059^***^ (−0.009)	−0.034^***^ (−0.007)	−0.077^***^ (−0.009)	−0.109^***^ (−0.017)	−0.058^***^ (−0.011)	−0.044^***^ (−0.005)	−0.076^***^ (−0.01)
*fukou*	0.232^**^ (−0.104)	0.018 (−0.262)	0.321^***^ (−0.105)	0.578^***^ (−0.22)	0.431 (−0.413)	0.682^***^ (−0.262)	0.242^**^ (−0.104)	0.638^***^ (−0.235)
*edu*	0.032 (−0.022)	−0.007 (−0.036)	0.060^**^ (−0.027)	0.059^*^ (−0.035)	−0.02 (−0.06)	0.110^**^ (−0.044)	0.034 (−0.023)	0.069^*^ (−0.037)
*marr*	0.006 (−0.037)	0.048 (−0.058)	−0.025 (−0.048)	−0.003 (−0.054)	0.062 (−0.087)	−0.041 (−0.07)	−0.008 (−0.038)	−0.007 (−0.056)
*inc*	0.048^***^ (−0.018)	0.057^*^ (−0.033)	0.045^**^ (−0.021)	0.057^*^ (−0.03)	0.04 (−0.052)	0.068^*^ (−0.037)	0.047^***^ (−0.018)	0.056^*^ (−0.031)
*heal*	−0.067^**^ (−0.026)	−0.06 (−0.051)	−0.069^**^ (−0.031)	−0.149^***^ (−0.045)	−0.105 (−0.084)	−0.165^***^ (−0.053)	−0.073^***^ (−0.027)	−0.169^***^ (−0.047)
*ill*	0.014 (−0.025)	0.037 (−0.049)	0.007 (−0.028)	0.067^*^ (−0.04)	0.127 (−0.078)	0.044 (−0.047)	−0.003 (−0.025)	0.052 (−0.042)
*child*	−0.018 (−0.021)	−0.001 (−0.042)	−0.025 (−0.025)	−0.021 (−0.037)	0.013 (−0.075)	−0.033 (−0.043)	−0.014 (−0.022)	−0.027 (−0.039)
*_cons*	3.470^***^ (−0.485)	4.590^***^ (−0.849)	2.840^***^ (−0.601)				3.693^***^ (−0.463)	
*cut1*				−4.657^***^ (−0.827)	−7.234^***^ (−1.463)	−3.210^***^ (−1.025)		−4.631^***^ (−0.837)
*cut2*				−3.443^***^ (−0.824)	−5.885^***^ (−1.453)	−2.043^**^ (−1.023)		−3.377^***^ (−0.836)
*cut3*				−2.805^***^ (−0.825)	−5.309^***^ (−1.454)	−1.376 (−1.024)		−2.734^***^ (−0.836)
*cut4*				−2.113^**^ (−0.828)	−4.754^***^ (−1.465)	−0.614 (−1.026)		−2.017^**^ (−0.839)
*cut5*				−0.789 (−0.833)	−3.419^**^ (−1.473)	0.704 (−1.032)		−0.74 (−0.843)
*N*	2,351	695	1,656	2,351	695	1,656	2,186	2,186
*r^2^*	0.064	0.075	0.064				0.07	
*F*	10.792	4.394	8.906				11.17	
*r2_p*				0.028	0.037	0.028		0.031
*Chi2*				144.462	59.594	106.835		150.959

Robustness standard errors in parentheses ^*^, ^**^, and ^***^ denote significance at 10%, 5%, and 1% levels.

The gender-specific regression analysis results are shown in Columns (2) and (3). The impact of perceived family relationships on the SPS of male UOALA failed the significance test, but the coefficient is greater than zero. In the female sample, the correlation between perceived family relationships and female UOALA remains evidently positive at the 5% level with a coefficient of 0.156, slightly lower than that of male UOALA.

The Ologit regression analysis results are shown in Columns (4)–(6). In the full sample estimation, the coefficient of family relationships (0.117) is evidently positive at the 5% level, which again supports hypothesis 1. In the test split by gender, the sample of male UOALA still failed the significance test, the correlation between perceived family relationships and female UOALA remains evidently positive at the 5% level with a coefficient of 0.123, which shows that female older adults are more sensitive to perceived family relationships.

The control variables are generally consistent with the theoretically expected results. Age, residency, income, and health factors all have a significant effect on the SPS of UOALA. The effect of age on SPS was significantly negative at the 0.01 level with a coefficient of −0.043, which indicates that the activeness in SPS of UOALA decreases with age, and that the decline in male UOALA's activeness in SPS is more evident. The residency variable has a positive effect at the 5% level, other things being equal, indicating that older adults with non-rural residency are more active in SPS. The effect of income level is evidently positive at the 0.01 level. Therefore, the higher the income of UOALA, the higher their activeness in SPS, and this is more pronounced in men. In addition, there is a positive correlation between the health of UOALA and their activeness in SPS, i.e., healthier UOALA prove to be more active.

### 3.2. Regional differences

To further explore the differential impact of cities, the region-specific sample regression was run, as shown in Table 3. Column (1) shows the sample of UOALA in first-tier cities (Shanghai and Guangzhou); column (2) shows the sample of UOALA in second-tier cities (Dalian and Chengdu); and column (3) shows the sample of UOALA in a third-tier city (Hohhot). The results suggest that there are regional differences in the effect of perceived family relationships on the SPS of older adults living alone. In first-tier and second-tier cities, a positive correlation exists between perceived family relationships and the SPS of UOALA at a 0.05 significance level, with coefficients of 0.255 in first-tier cities and 0.229 in second-tier cities, which are both higher than the benchmarking regression coefficient of 0.170; the effect in third-tier cities is not as significant, with a small coefficient of 0.024. This suggests that the higher the degree of urban socioeconomic development, the stronger the influence of perceived family relationships on the SPS of UOALA.

**Table 3:** Effects of perceived family relationships on SPS in different classes of cities.

	**The predicted variable:** ***soc*** **(social participation through sports)**					
	**Benchmarking regression**			**Robustness test**		
	**First-tier cities**	**Second-tier cities**	**Third-tier cities**	**First-tier cities**	**Second-tier cities**	**Third-tier cities**
	**(1)**	**(2)**	**(3)**	**(4)**	**(5)**	**(6)**
*fam*	0.255^**^	0.229^**^	0.024	0.140^**^	0.191^***^	0.125
	−0.105	−0.095	−0.098	−0.067	−0.07	−0.113
Control variables	Control	Control	Control	Control	Control	Control
*N*	1,031	894	426	920	842	424
*r2*	0.057	0.053	0.104	0.064	0.06	0.104
*F*	6.495	4.17	6.698	6.217	4.793	6.367

Robustness standard errors in parentheses ^*^, ^**^, and ^***^ denote significance at 10%, 5%, and 1% levels.

### 3.3. Robustness tests

To ensure the reliability of the findings of the benchmarking regression analysis, the self-rated difficulty in response to the question “As you age, do you think it is difficult in communicating with your children or grandchildren?” was used as a proxy variable (“Yes = 1; A little = 2; No = 3”) for the variable of perceived family relationships. Columns (7) and (8) in Table 2 show the results of the robustness test. According to both OLS model estimation and Ologit model estimation, a positive correlation exists between perceived family relationships and the SPS of UOALA at a 0.05 significance level, which still supports hypothesis 1. Similarly, columns (4)–(6) in Table 3 show the results of robustness tests in different cities. Other things being equal, a positive correlation exists between perceived family relationships in first-tier cities and the SPS of UOALA at a 0.05 significance level, with a coefficient of 0.140; perceived family relationships in second-tier cities have a positive effect at a 0.01 significance level, with a coefficient of 0.191; and the effect of family relationships in third-tier cities remains insignificant, which shows that the results of this paper are robust.

### 3.4. Endogeneity

There are mainly four causes of endogeneity: omitted variable, selection, self-selection bias, sample selection bias and simultaneity. An instrumental variable two-stage regression model was used to effectively address the endogeneity problem and thus more accurately identify the effect of perceived family relationships on the SPS of UOALA. Specifically, the selected instrumental variable should be highly correlated with the substituted endogenous variables, but independent of the random error term. Therefore, the “parent-child residential proximity” (prox) was selected as an instrumental variable. The progress of modernization has brought about changes in individual cognition, family demographics, etc., thus leading to the looseness of the traditional family structure. Intergenerational living reflects the organization of family life and the way family members interact (32).

According to the theory of intergenerational solidarity, intergenerational living can motivate each other to provide financial, caring and emotional support between generations, and positively improve the wellbeing of family members (33). Since the study focused on older adults living alone in urban areas, cases of intergenerational living were excluded, but parent-child residential proximity is still an important measure of intergenerational living conditions. The closer the proximity, the higher the frequency of intergenerational interactions, and the higher the likelihood of achieving harmonious perceived family relationships. Therefore, the variable substitution was based on the “parent-child residential proximity”: in the same neighborhood = 1; in the same street or town but a different neighborhood = 2; in the same city (district or county) but different streets or towns = 3; in the same province (autonomous region or municipality directly under the Central Government) but different cities (districts or counties) = 4; in the Chinese mainland, but different provinces (autonomous regions or municipalities directly under the Central Government) = 5; outside Chinese mainland = 6.

The instrumental variables were estimated using the “two-stage least squares” method, as shown in Table 4. In the first stage, the OLS method was used to run a regression of the instrumental variables on the endogenous explanatory variables, with perceived family relationships as the dependent variable and regressing the instrumental variables on the other control variables. In the second stage, the true values were replaced by the predicted values of perceived family relationships in the first stage and then the regression was run. The Hausman test was performed with a *p*-value of 0.0000 (<0.05) for the full sample, rejecting the null hypothesis that all variables were exogenous. And the instrumental variables approach should be used. Since the traditional Hausman test was invalid under heteroskedasticity, the heteroskedasticity-robust Durbin test and Wu-Hausman test were performed with *p*-values of 0.0062 (<0.05) and 0.0063 (<0.05), respectively, rejecting the null hypothesis that all variables were exogenous; meanwhile, the instrumental variables passed the weak instrumental variable test.

**Table 4:** Instrumental variables regression of perceived family relationships on SPS.

	**The predicted variable:** ***soc*** **(social participation through sport)**		
	**Full sample**	**Male**	**Female**
	**(1)**	**(2)**	**(3)**
*fam*	2.177^***^	3.063^*^	1.734^*^
	−0.801	−1.724	−0.928
Control variables	Control	Control	Control
Cities	Control	Control	Control
*N*	2,347	694	1,653
*chi2*	116.855	30.789	91.933
**First-stage regression**			
*prox*	−0.040^***^	−0.041^**^	−0.038^***^
	−0.009	−0.018	−0.01
Control variables	Control	Control	Control
Cities	Control	Control	Control
*F*	15.491	6.568	10.634

Robustness standard errors in parentheses ^*^, ^**^, and ^***^ denote significance at 10%, 5%, and 1% levels.

The estimates of the full sample are shown in Column (1). According to the first-stage regression, the intergenerational residential proximity correlates significantly with perceived family relationships of UOALA at the 0.01 level, i.e., the closer the intergenerational residential proximity, the better the relationship between UOALA and other family members. According to the estimated results of the second stage, a significant positive correlation exists between perceived family relationships and the SPS of UOALA, with a coefficient (2.177) higher than the estimated coefficient (0.170) from the benchmarking regression. It suggests that the estimation without instrumental variables may lead to a high degree of underestimation. Gender-specific estimates are shown in columns (2) and (3). According to the first-stage regression, a significant positive correlation exists between intergenerational residential proximity and perceived family relationships of both male and female UOALA. The second-stage regression shows a decrease in significance for both gender-specific samples compared to the full sample, but the coefficient of the men's sample is higher than that of the full sample and women's sample. Perceived family relationships have a greater effect on the SPS of male UOALA, with coefficients that are higher than the benchmarking regression results, and estimation without instrumental variables similarly may lead to a high degree of underestimation.

### 3.5. Mediation effect analysis

So far, this paper has focused on the effect of perceived family relationships on the SPS of UOALA. This section will discuss the mediating factor of this effect and the mechanism behind it. Based on the hypothesis mentioned above, it is speculated that perceived family relationships may indirectly affect the SPS of UOALA by influencing their self-respect levels.

The estimates of the level of self-respect as a mediating variable are shown in Table 5. The overall estimated results are shown in columns (1)–(3). The results in column (1) show that a significant positive correlation exists between perceived family relationships and the SPS of UOALA, with a coefficient of 0.170, indicating that the better the family relationship of UOALA, the higher the activeness in SPS. The results in column (2) show that a significant positive correlation exists between perceived family relationships and the self-respect level of UOALA, i.e., The better the perception of family relationship, the higher the level of self-respect. According to column (3) where the effects of perceived family relationships and self-respect levels on SPS were studied at the same time, self-respect level has a positive effect on SPS, and the effect of perceived family relationships on SPS is no longer significant with the coefficient becoming smaller. Thus, self-respect levels play a major mediating role in the influence of perceived family relationships on SPS. As a result, hypothesis 3 is supported.

**Table 5:** Tests of the mediating role of self-respect levels in the effect of perceived family relationships on the SPS of UOALA.

	**Full sample**			**Male**			**Female**		
	***soc***	***resp***	***soc***	***soc***	***resp***	***soc***	***soc***	***resp***	***soc***
	**(1)**	**(2)**	**(3)**	**(4)**	**(5)**	**(6)**	**(7)**	**(8)**	**(9)**
*fam*	0.170^***^	0.070^*^	0.118	0.202^**^	0.042	0.162	0.156^**^	0.093^*^	0.085
	−0.058	−0.039	−0.073	−0.102	−0.066	−0.112	−0.07	−0.048	−0.094
*resp*			0.142^***^			0.1			0.161^***^
			−0.051			−0.1			−0.059
*_cons*	3.470^***^	2.144^***^	3.304^***^	4.590^***^	2.411^***^	4.200^***^	2.840^***^	1.917^***^	2.791^***^
	−0.485	−0.287	−0.588	−0.849	−0.492	−0.997	−0.601	−0.355	−0.753
*N*	2,351	1,773	1,744	695	543	535	1,656	1,230	1,209
*r2*	0.064	0.262	0.069	0.075	0.307	0.078	0.064	0.245	0.072
Control variables	Control	Control	Control	Control	Control	Control	Control	Control	Control
Cities	Control	Control	Control	Control	Control	Control	Control	Control	Control
*F*	10.792	54.485	8.497	4.394	22.783	3.605	8.906	39.451	6.825

Robustness standard errors in parentheses ^*^, ^**^, and ^***^ denote significance at 10%, 5%, and 1% levels.

Gender-specifically, the estimated results of the men's sample are shown in columns (4)–(6). The results in column (4) indicate that perceived family relationships have a positive impact on the SPS of UOALA at the 0.05 significance level, with a coefficient of 0.202. The results in column (5) indicate that the impact of perceived family relationships on self-respect levels failed the significance test. In column (6), the variables of perceived family relationship and self-respect levels were substituted at the same time. The results show that both have no significant effect, but the coefficient of perceived family relationships (0.162) is lower than the estimate in column (4). It follows that the level of self-respect plays a mediating role (not significant) in the effect of perceived family relationships on the SPS of male UOALA. The estimated results of the female sample are shown in columns (7)–(9). According to column (7), a significant positive correlation exists between perceived family relationships and the SPS of female UOALA at a 0.05 significance level, with a coefficient of 0.156. The results in column (9) show that the level of self-respect has a significant positive effect at the 0.01 level and the effect of perceived family relationships is no longer significant, with a decreased coefficient of 0.085. This is consistent with the estimated results of the full sample, i.e., the level of self-respect plays a significant mediating role in the effect of perceived family relationships on the SPS of female UOALA.

## 4. Discussion

The purpose of this study is to explore the influence of family relationship perception of UOALA on SPS and find out the mechanism. The results show that the perceived family relationship has a positive impact on the sports social behavior of the older adults living alone in the city, that is, the better the perceived family relationship, the higher the sports social activity of them. The quality of life of the older adults depends on their family environment, and the acquisition of health welfare and happiness is largely controlled by family members (34). Similarly, the intensity of the intergenerational relationship had a significant effect on exercise behavior (35). The intergenerational relationship explained by the intergenerational solidarity theory just provides an explanation for the influencing factors of social participation through sports of the older adults from the micro level. Meanwhile, in the sub-sample test, it is found that the perception of family relationship of female older adults has a stronger promoting effect on their SPS. Given the fact that women's life expectancy is higher than men's. SPS is not only an effective way for female seniors living alone to build health and prevent the aggravation of diseases, but also a platform to re-establish social connections for older adults. Considering that women are at greater risk of living alone in their later years, the life-long SPS not only relieve their social pressure, but also can prevent them from succumbing to traditional gender roles to a certain extent, especially when the gender order still plays a part, thus enhancing the identification of new gender roles.

In addition, the data results of control variables also show that different accumulation levels of individual capital affect the differentiation in SPS. The different accumulation levels of economic capital, health capital, and cultural capital have an impact on the scope of the SPS of UOALA and their persistence, and such distinction amounts to social stratification in the field of SPS.

In the analysis of regional differences, we found that family relationship perception has a more significant impact on the older adults living alone in the first and second tier cities. Rapid socio-economic development has resulted in historical fragmentation at the macro level and physical isolation at the micro-level, which has tangibly or invisibly detached individuals from social “shared experiences” and increased the likelihood of their existence as “atomized” individuals (36). Due to the weakening of the community space as a social reference system for residents to identify with each other, the lasting sense of belonging that has been formed over a longtime fades away. The alienation of relationships weakens both the social and public attributes of the community, which is more evident in economically developed cities (37). The frequent movement of people in large cities and the volatility and instability of urban space increase the uncertainty and even risks faced by individuals (38).

Older adults are more susceptible to physical and psychological factors, and thus need more time for social adaptation. However, the special state of living alone makes it difficult for them to adapt to the ever-changing social environment in a limited and short period. As a result, they are more likely to seek a safer way of social interaction, choosing to retreat from the noisy and changing public sphere into the relatively quiet and isolated space of the family. Only when the family space can give them sufficient psychological support and positive feedback will they be “confident” enough to engage in more complex social activities and be more active in SPS. The social modernization and high level of urbanization have led to the alienation of social relationships and the atomization of social structures. Due to the increasingly prominent cognition of value based on families and even individuals, families have the responsibility to motivate more older adults to be active in SPS.

Finally, in the test of mediating effect, we found that perceived family relationship affects SPS of older adults living alone through self-respect level. Self-respect is an important part of the self-system. It is about an individual's positive or negative self-evaluation, reflecting a subjective need for a sense of self-worth and societal acknowledgment. A high level of self-respect can help improve individuals' adaptability and survivability. Positive family relationships lead to positive emotional experiences as well as a more positive evaluation of self-worth, which may increase the likelihood of SPS in old age.

This study has the following limitations. First, this study is based on the analysis of cross-sectional data. The survey objects are older adults living alone for more than half a year at the time of the survey. Therefore, in the subsample regression of age, the relevant classification refers to the actual age at the time of the survey, rather than the cohort data of the follow-up survey. Second, the data used in this study are large social surveys conducted by university research teams which funded by the government. Due to the difficulty in obtaining such large-scale micro survey data, it is a pity that we cannot obtain latest relevant authoritative data. If future data conditions permit, we will use the updated data for follow-up investigation of this study.

## 5. Conclusions

Changing times and social development have brought about new changes in the social relationships and functions faced by older adults living alone in urban areas. The increasing complexity of the SPS of UOALA due to the changes in social environments and the size and structure of families intertwined with changing behavior and mindsets of the older adults deserves a reexamination. In this study, regression model and mediation effect analysis were used to study the relationship between perceived family relationship and social participation through sports of older adults living alone, as well as the mediating path between them. The results show that there is a significant relationship between the perceived family relationship and social participation through sports of the older adults living alone, and the level of self-respect also plays an intermediary role in this relationship.

In China, emotional support, as an intrinsic function and core attribute of the family, has not been completely weakened or eliminated during the short-term reconfiguration of society. Even when parents and children live in different places, if children stay in close touch with parents and provide emotional support, it will promote their activeness in SPS. From the perspective of social intervention, to improve their activeness in SPS, we can use family relationships as an entry point in order to help older adults build their self-worth and self-respect.

Therefore, families should actively encourage lone parents to build social connections through sport. When the older adults retire, their scope of life is often limited to family and community, and interpersonal interactions are mainly with family members and relatives. The weakening of social ties at the workplace has reduced the opportunities for the older adults living alone to socialize with others, leading to a gradually shrinking social network size and even triggering social phobia in them. To address the problem, family members can help parents rebuild self-respect and self-confidence by encouraging them to engage in sporting activities, thus making them aware of their social role and stimulating their activeness in SPS.

## Data availability statement

The original contributions presented in the study are included in the article/supplementary material, further inquiries can be directed to the corresponding author.

## Author contributions

Methodology: XXY. Writing original draft preparation and writing review and editing: JHC, XXY, and RZ. Funding acquisition: RZ. All authors have read and agreed to the published version of the manuscript.
